# Identification of biomarkers for hepatocellular carcinoma using network-based bioinformatics methods

**DOI:** 10.1186/2047-783X-18-35

**Published:** 2013-10-01

**Authors:** Lingyan Zhang, Ying Guo, Bibo Li, Juan Qu, Chunbao Zang, Fang Li, Ying Wang, Hua Pang, Shaolin Li, Qingjun Liu

**Affiliations:** 1 Department of Prevention and health care, Mianyang Central Hospital, No.12 Changjia Alley, Fucheng District, Mianyang, Sichuan 621000, P.R. China; 2 Department of Radiology, College of Basic Medicine, Chongqing Medical University, No.1 Yixueyuan Road, Yuzhong District, Chongqing 400016, P.R. China; 3 Department of Oncology, The Third People’s Hospital of Chongqing, Chongqing 400014, P.R. China; 4 Department of otolaryngology, Xijing Hospital, Fourth Military Medical University, Xi’an 710032, Shaanxi Province, P.R. China; 5 Department of Radiation Oncology, Chongqing Cancer Institute/Hospital, No.181 Hanyu Lane, Shapingba District, Chongqing 400030, P.R. China; 6 Department of Nuclear Medicine, the First Affiliated Hospital of Chongqing Medical University, No.1 Youyi Road, Yuzhong District, Chongqing 400016, P.R. China; 7 Department of otolaryngology, Mianyang Central Hospital, No.12 Changjia Alley, Fucheng District, Mianyang, Sichuan 621000, P.R. China

**Keywords:** Hepatocellular carcinoma, Biomarker, Protein-protein interaction

## Abstract

**Background:**

Hepatocellular carcinoma (HCC) is one of the most common types of cancer worldwide. Despite several efforts to elucidate molecular mechanisms involved in this cancer, they are still not fully understood.

**Methods:**

To acquire further insights into the molecular mechanisms of HCC, and to identify biomarkers for early diagnosis of HCC, we downloaded the gene expression profile on HCC with non-cancerous liver controls from the Gene Expression Omnibus (GEO) and analyzed these data using a combined bioinformatics approach.

**Results:**

The dysregulated pathways and protein-protein interaction (PPI) network, including hub nodes that distinguished HCCs from non-cancerous liver controls, were identified. In total, 29 phenotype-related differentially expressed genes were included in the PPI network. Hierarchical clustering showed that the gene expression profile of these 29 genes was able to differentiate HCC samples from non-cancerous liver samples. Among these genes, *CDC2* (*Cell division control protein 2 homolo*g), *MMP*2 (*matrix metalloproteinase-2*) and *DCN* (*Decorin* were the hub nodes in the PPI network.

**Conclusions:**

This study provides a portfolio of targets useful for future investigation. However, experimental studies should be conducted to verify our findings.

## Background

Hepatocellular carcinoma (HCC), a primary liver cancer, is the fifth most common cancer worldwide and the third most common cause of cancer mortality [1]. An estimated 748,300 new liver cancer cases and 695,900 cancer deaths occurred worldwide in 2008 [2]. This disease is most prevalent in eastern and southeastern Asia, and in middle Africa, with more than half of patients with HCC being reported from China [3]. In addition, evidence has been accumulating in various countries that the incidence of HCC is rising [4-7]. To improve treatment and prognosis of HCC, information about the phenotypic and molecular changes associated with the development of this disease should be determined.

Much is known about the causes and development of HCC. The main causative agents, hepatitis B virus (HBV), hepatitis C virus (HCV), and aflatoxin B1, together account for about 80% of all HCCs in humans [1,8-11]. Hepatocarcinogenesis is a complex process associated with the accumulation of genetic and epigenetic changes that occur during initiation and progression of the cancer. In recent years, a number of genomic studies have identified genes that are uniquely upregulated or downregulated in HCC tissues. For example, Lee *et al*. suggested that cystatin B (*CSTB*) or the combination of *CSTB* and α-fetoprotein may be useful markers for diagnosis with high sensitivity of patients with HCC [12]. In addition, potential biomarkers for detection of early HCC [13], such as glypican 3 (*GPC3*) [14], ADAM metallopeptidase domain 12 (*ADAM12*) [15], serine/threonine kinase 15 (*STK15*), phospholipase A2 (*PLA2*) [16], and heat-shock protein 70 (*HSP70*) [17] have also been suggested by previous studies. However, despite several previous efforts, the current understanding or early diagnosis of HCC is still rather limited.

The advancement of microarray technology now enables elucidation of the molecular mechanism of HCC development and identification of novel diagnostic biomarkers. In this study, to acquire further insights into the molecular mechanisms of HCC, we downloaded gene expression profiles of 10 HCCs and 10 noncancerous liver controls from the Gene Expression Omnibus (GEO) database, and analyzed those data using bioinformatics tools. We identified a set of interactive genes that were significantly downregulated or upregulated in HCC. These data may help to improve the diagnostic accuracy of HCC.

## Methods

### Microarray data

The gene expression profiles of HCC with non-cancerous liver controls, which were deposited by Deng and colleagues (accession number: GSE19665,) (approved by ethics committee of Mianyang Central Hospital) were downloaded from GEO [18]. The mRNA expression in ten HCCs (five HBV-related and five HCV-related HCCs) and the 10 matched non-cancerous liver samples (five HBV-related and five HCV-related chronic hepatitis or cirrhosis) was analyzed byoligonucleotide arrays (GeneChip Human Genome U133 plus 2.0; Affymetrix Inc., Santa Clara, CA, USA). For global normalization, the average signal in an array was made equal to 100. We downloaded the raw CEL data and the annotation file for the platform.

### Protein-protein interaction data

A total of 36,289 pairs of protein-protein interactions (PPIs) were downloaded from the Human Protein Reference Database (HRPD; http://www.hprd.org/) [19] in March, 2011. Of these, 34,704 pairs of PPIs have relationships with expression profiles. Data preprocessing and identification of differentially expressed genes.

The Affy package in R [20,21] was used to preprocess the raw expression data. We first converted the probe-level data in the CEL files into expression measures. For each sample, the expression values of all probes for a given gene were reduced to a single value by taking the average expression value; this yielded a set of 19,803 genes. The Significance Analysis of Microarrays (SAM) software [22] was used to identify differentially expressed genes (DEGs). We considered a false discovery rate (FDR, corrected by the Benjamini and Hochberg method [23]) of less than 0.01 to be significant.

### Functional enrichment tests

The Kyoto Encyclopedia of Genes and Genomes (KEGG) pathway database records networks of molecular interactions in the cells, and variants of these interactions specific to particular organisms [24]. To explore the dysfunctional pathways in HCC, we inputted the candidate genes into the Database for Annotation, Visualization, and Integrated Discovery (DAVID; http://david.abcc.ncifcrf.gov/) for pathway enrichment analysis. DAVID is a web-based software suite designed to categorize complex, high content, genomic and proteomic datasets [25]. FDR <0.05 was selected as the cut-off criterion.

### Construction of the PPI network

First, we identified phenotype-related genes by calculating the Pearson correlation coefficient (*r*). The genes that showed significant correlation with HCC (*r* >0.8 or *r* < −0.8) were selected as phenotype-related genes. The phenotype-related genes and DEGs were then intersected to obtain the phenotype-related DEGs. Meanwhile, we filtered the significant PPIs in the HPRD database with a cut-off criterion of *r* >0.8 or *r* < −0.8. Finally, we mapped the phenotype-related genes for HCC to the significant PPIs, and constructed a PPI network using Cytoscape software [26].

## Results

### Identification of DEGs

The gene expression profile of GSE19665 was downloaded from the GEO database and theSAM method was used to identify DEGs in HCC compared with non-cancerous controls. At FDR <0.01, 2,767 genes were identified as DEGs. Of these, 1,359 genes (49.11%) were upregulated and the remaining 1,408 genes (50.89%) were downregulated.

### Functional enrichment tests

To functionally classify these 2,767 significant genes, we used the online biological classification tool DAVID, and found significant enrichment of these genes in three pathways (Table 1). The most significant pathway was the cell cycle with FDR = 0.0130. The other significant pathways were complement and coagulation cascades (FDR = 0.0214) and DNA replication (FDR = 0.0251).

**Table 1:** The enriched pathways for differentially expressed genes (FDR < 0.05)

**Pathway ID**	**Pathway name**	**Gene count**	***P***	**FDR**
**hsa04110**	Cell cycle	121	1.37E-04	0.0130
**hsa04610**	Complement and coagulation cascades	67	1.13E-04	0.0214
**hsa03030**	DNA replication	36	3.99E-04	0.0251

Further, we performed pathway enrichment analysis separately for the upregulated and downregulated genes. The 1,359 upregulated genes were enriched to 12 pathways (Table 2), including cell cycle, DNA replication, base excision repair, and nucleotide excision repair, while the 1,408 downregulated genes were enriched to 9 pathways (Table 3), including complement and coagulation cascades, chemokine signaling pathway, and cytokine-cytokine receptor interaction.

**Table 2:** The enriched pathways for up-regulated genes (FDR< 0.05)

**Pathway ID**	**Pathway name**	**Up genes**	***P***	**FDR**
**hsa04110**	Cell cycle	36	1.08E-11	1.78E-09
**hsa03030**	DNA replication	17	5.07E-09	4.16E-07
**hsa03050**	Proteasome	14	1.80E-05	9.82E-04
**hsa03410**	Base excision repair	12	3.70E-05	0.0015
**hsa03420**	Nucleotide excision repair	13	1.50E-04	0.0049
**hsa00970**	Aminoacyl-tRNA biosynthesis	12	3.31E-04	0.0090
**hsa04120**	Ubiquitin mediated proteolysis	24	3.43E-04	0.0080
**hsa03430**	Mismatch repair	8	0.0014	0.0280
**hsa03440**	Homologous recombination	9	0.0014	0.0250
**hsa04114**	Oocyte meiosis	19	0.0016	0.0256
**hsa03040**	Spliceosome	21	0.0020	0.0292
**hsa04914**	Progesterone-mediated oocyte maturation	16	0.0024	0.0323

**Table 3:** The enriched pathways for down-regulated genes (FDR < 0.05)

**Pathway ID**	**Pathway name**	**Down genes**	***P***	**FDR**
**hsa04610**	Complement and coagulation cascades	27	1.37E-09	2.31E-07
**hsa04062**	Chemokine signaling pathway	43	2.53E-07	2.14E-05
**hsa04060**	Cytokine-cytokine receptor interaction	54	4.37E-07	2.46E-05
**hsa04640**	Hematopoietic cell lineage	24	9.55E-06	4.03E-04
**hsa00590**	Arachidonic acid metabolism	17	6.48E-05	0.0022
**hsa05020**	Prion diseases	12	5.63E-04	0.0157
**hsa05340**	Primary immunodeficiency	12	7.43E-04	0.0178
**hsa04672**	Intestinal immune network for IgA production	14	7.84E-04	0.0164
**hsa04510**	Focal adhesion	35	0.0026	0.0484

### Construction of PPI network

In total, 314 phenotype-related genes were identified with *r* > 0.8 or *r* < −0.8. Most of these genes were DEGs between HCCs and noncancerous liver samples, except for *ISCA2* (iron-sulfur cluster assembly 2 homolog).

There were 399 pairs of PPIs filtered from HPRD with *r* > 0.8 or *r* < −0.8. By mapping the phenotype-related DEGs to these PPI data, we obtained 24 pairs of PPIs, including 29 nodes (Figure 1). We found that *CDC2* (*Cell division control protein 2 homolo*g), *MMP*2 (*matrix metalloproteinase-2*) and *DCN* (*Decorin*) were hub nodes in the PPI network, suggesting that these genes may play important role in the initiation of HCC.

**Figure 1:** ***CDC2*, *MMP2*, and *DCN *** **are hub nodes in the protein-protein interaction (PPI) network constructed by phenotype related differentially expressed genes (DEGs).**

### Hierarchical clustering

To verify whether the 29 genes in the PPI network could be used to differentiate between HCC and non-cancerous liver, we performed hierarchical clustering using R based on gene expression level (Figure 2). We found that although the 29 gene profiles could notdifferentiate HCV-related HCCs from HBV-related HCCs, they could differenttiate HCC samples from non-cancerous livers. In addition, hierarchical clustering portioned the genes into two groups. In total, 15 genes were upregulated in HCC, including *THBS1* (Thrombospondin 1), *IGFBP3* (insulin-like growth factor binding protein 3), *GPRASP1* (G protein-coupled receptor associated sorting protein 1), *DPT* (dermatopontin), and *MMP2*. The other 14 genes were downregulated in HCC, and included *TUBG1* (tubulin, gamma 1), *CDKN2C* (Cyclin-dependent kinase 4 inhibitor C), *CDKN2A* and *RRM2* (ribonucleotide reductase M2).

**Figure 2:** **Hierarchical clustering of genes in the protein-protein interaction (PPI) network.** Rows represent genes and columns represents sample. The samples under the green bar were noncancerous liver samples and the samples under the purple bar were hepatocellular (HCC) samples.

## Discussion

Although previous studies have generated a large number of biomarkers for early diagnosis of HCC, the efficiency of current therapy of patients with this disease is still low. In addition, the molecular mechanism of HCC is still not fully understood. In this study, we analyzed the gene expression profile of HCC and non-cancerous liver samples using a combined bioinformatics approach. The dysregulated pathways and PPI network, including hub nodes that distinguished HCCs from noncancerous liver controls, were identified.

Our approach identified an HCC molecular signature of 29 genes. Hierarchical clustering showed that the gene expression profile of these 29 genes was able to differentiate HCC samples from noncancerous livers. Of these genes, *CDC2*, *MMP2*, and *DCN* were hub nodes in the PPI network. Studies suggest that more centralized genes in the network are more likely than peripheral genes to be key drivers of proper cellular function [27].

CDC2, also known as CDK1, is a member of the serine/threonine protein kinase family. This protein is a catalytic subunit of the highly conserved protein kinase complex known as M-phase promoting factor, which is essential for G1/S and G2/M phase transitions of the eukaryotic cell cycle. In our study, CDC2 was differentially expressed in HCC compared with noncancerous lives. A previous study suggested that CDC2 plays the most crucial role of the G2/M modulators in cell cycle progression and cell proliferation of HCC, and significantly predicts the recurrence of this carcinoma [28]. Another study showed that CDC2 and CDK2 are activated in HCC, and this may be due to a complex interplay between the level of cyclin, CDK, CDK inhibitors, and inhibitory phosphorylation [29]. In accordance with this study, our PPI network showed that CDC2 directly interacted with CCNB1, CCNB2, and CDKN3. In addition, FOXM1 (Forkhead box protein M1), TOP2A, RRM2, and ECT2 were also identified as having interactions with CDC2. FOXM1 is a human cell cycle transcription factor that is known to play a key role in regulating timely mitotic progression and chromosomal segregation during cell division [30]. Xia *et al*. reported that activation of FOXM1 through the ERK/CREB pathway is involved in HBV-related hepatocarcinogenesis [31]. Overexpression of TOP2A was reported to be correlated with earlier onset, shorter survival time, and resistance to chemotherapy in HCC [32]. RRM2 is located in a region of frequent cytogenetic aberration in HCC [33]. Chua *et al*. suggested that gallium maltolate might be a promising chemotherapeutic agent for treatment of HCC by targeting RRM2 [34].

MMP2 is a key member of the matrix metalloproteinase (MMP) family, which is involved in many pathological conditions, particularly cancer metastasis and angiogenesis [35,36]. Our result suggested that MMP2 is upregulated in HCC, and this result is in line with previous studies [37-41]. The PPI network in our study showed that MMP2 directly interacted with six DEGs: TIMP2, CXCL12, DCN, FGFR1, THBS1, and IGFBP3. TIMP2 is the tissue inhibitor of MMP2. An imbalance between the proteolytic activity of MMP2 and TIMP2 is responsible for degradation of extracellular matrix (ECM) components, and plays a crucial role in tumor invasion and in metastasis formation [42]. Theret *et al*. also found a correlation between MMP mRNA levels and MMP2 and TIMP2 mRNA levels, as well as with MMP2 activation in HCCs [43]. THBS1 is a matricellular protein capable of modulating angiogenesis, and high expression of THBS1was shown to be associated with tumor invasiveness and progression in HCC [44]. IGBP-3 is a mediator of growth suppression signals and a putative tumor suppressor. It was reported that IGFBP-3 mediates growth suppression signals via the transforming growth factor-β and/or Rb pathways in HCC [45].

DCN is a small cellular or pericellular matrix proteoglycan that is closely related in structure to biglycan protein. Our result suggested that DCN is differentially expressed in HCC and interacts with DPT, THBS1, MMP2 and COL14A1. Few studies have reported DCN expression in HCC, therefore its potential role in hepatocarcinogenesis remains to be investigated. In addition, increased expression levels of S100A8 and S100A9 have been detected in various human cancers in recent years [46]. Nemeth *et al*. suggest that S100A8 and S100A9 are novel nuclear factor-κB target genes in HCC cells, and increased expression of these proteins supports malignant progression by activation of reactive oxygen species-dependent signaling pathways [47].

There are some limitations to our study. First, we did not generate the microarray data ourselves but took them from the GEO database. Second, as differences exist between HBV-related and HCV-related cancers, elaboration of HBV-specific or HCV-specific genes may be more important. Third, validation of the results in other datasets or samples is lacking in this study, therefore, further experimental studies based on a larger sample size are needed to confirm our results. This would be the next step in our research.

## Conclusion

In conclusion, we have identified an HCC molecular signature of 29 genes. Of these genes, *CDC2*, *MMP2*, and *DCN* were hub nodes in the PPI network. However, further experimental studies are necessary to confirm our results and to elucidate the role of these genes in HCC pathogenesis and to determine their potential as molecular targets for the development of new therapeutic approaches for HCC.

## Competing interests

The authors declare that they have no competing interests.

## Authors’ contributions

LYZ and YG Conceived and designed the experiments; BBL,and JQ Analyzed the data. CBZ and FL Contributed reagents/materials/analysis tools; YW,HP,SLL and QJL Wrote the paper. All authors read and approved the final manuscript.

## Authors’ information

Lingyan Zhang and Ying Guo should be regarded as co-first authors.
